The article "Application of CFD Numerical Simulation Image Imaging Technology in the Study of Droplet Microfluidic Multiphase Flow Characteristics" was retracted in 2023. Reasons: suspected computer-generated content; unreliable results or conclusions; concerns about the data; concerns about the results or conclusions.

# Application of CFD Numerical Simulation Image Imaging Technology in the Study of Droplet Microfluidic Multiphase Flow Characteristics

**DOI:** 10.1155/2022/5851658

**Published:** 2022-06-27

**Authors:** Hao Li, Zihan Hu

**Affiliations:** Central South University, Changsha, Hunan 410000, China

## Abstract

In order to study the problem that the flow in the internal channel of the microfluidic chip is different from that of the macroscopic system by the FD numerical simulation image imaging technology. Taking the liquid-liquid extraction of microfluidic chip as the research object, this paper analyzes the theoretical basis, working principle, structural parameters, and the influence of working parameters on the fluid flow of liquid-liquid extraction. The results are as follows: when the inlet velocity of flowing liquid is 10^^(−5)^ m/s, the diffusion efficiency can still be maintained at 95%; the double *ψ*-type aqueous phase showed laminar flow, the two-phase contact interface increased compared with the bottom flow rate, and the extraction efficiency increased to 98%; the extraction efficiency of double *ψ* type is higher than that of double Y-type: when the flow velocity ratio increases from *v*_*aq*_ : *v*_oil_=1 : 2 to *v*_*aq*_ : *v*_oil_=5 : 1, the extraction efficiency increases to 99.8%; the experimental extraction efficiency is compared with the diffusion efficiency simulated by simulation. The diffusion efficiency of the cross type is 1.05 times that of the extraction efficiency, and that of the cylindrical type is 1.04 times that of the extraction efficiency. In this study, CFD is used to simulate the characteristics of droplet microfluidic multiphase flow, which enriches the theoretical method and research experience of liquid-liquid laminar flow.

## 1. Introduction

Process strengthening is the key technology to realize the green process. Through the development of small-size and miniaturized equipment, the unit energy consumption and by-product generation are reduced, and finally the purpose of improving production efficiency, reducing production cost, improving safety, and reducing environmental pollution is achieved. However, the development of small and compact equipment also brings new challenges to the research of hydrodynamic characteristics and motion behavior, especially in multiphase flow system. Compared with the traditional macro large-scale system, the two-phase fluid controlled by microchannel has the advantages of large specific surface area, short transfer distance, and fast mixing speed. It can reduce the mass transfer limitation and obtain better performance. Therefore, liquid-liquid microfluidic systems have made great progress in the fields of chemical reaction, liquid-liquid extraction, bioanalysis, crystallization process regulation, and the preparation of structural materials. In order to analyze the effects of operating conditions, fluid properties, and channel structure on multiphase flow, many useful studies have been carried out from the perspective of experiment [1].

According to previous experimental studies, the interaction and dynamic behavior of two-phase flow in microchannel are affected by many parameters, such as two-phase velocity, two-phase viscosity, interfacial tension, microchannel structure, and wall wetting characteristics. At the same time, the theoretical analysis of predicting droplet size and forming mechanism in microchannel device is still complex and inaccurate. Therefore, it is difficult to fully understand the phenomenon and characteristics of two-phase flow in microchannels only by experimental research or theoretical analysis. At the same time, the measurement of parameters and the acquisition of flow field characteristics in microfluidic system are also very difficult. Due to these two reasons, the current microfluidic system theory is mostly empirical research [2].

In addition, the motion of droplets and bubbles in complex geometry is very important for many scientific and engineering applications. In the past decades, the movement of bubbles and droplets in unconstrained media has attracted great attention in the scientific community. On the contrary, the research on the evolution of bubble droplets in complex geometric channels is very limited (Figure 1). On the one hand, the microchannel wall can compress bubbles and droplets. To some extent, the shape of droplets/bubbles is determined by the microchannel structure. On the other hand, bubbles/droplets can evolve freely in unbounded media but move under the restriction of microchannel structure. In order to study these two kinds of phenomena, we usually separate them from the macroscopic process. For the evolution of droplets or bubbles in complex geometry, some approximate analytical solutions are obtained by simplifying the governing equation. Therefore, it is very necessary to develop numerical simulation methods that can realize complex mass and heat transfer processes such as droplet forming, droplet coalescence/fusion, droplet dissolution, and particle focusing in microchannels [3].

## 2. Literature Review

Vollertsen et al. believe that the development and application of microfluidic technology have developed vigorously in recent years, but the basic theoretical research on flow mechanism and liquid-phase mass transfer in microchannels is not sufficient, especially for the theoretical research and experimental conclusions of multiphase liquid-liquid microextraction technology, there have been few research results at home and abroad in recent years [4]. Xie et al. believe that liquid-liquid extraction technology, as a common means in chemical analysis and detection, in the microfluidic chip, because the use of most extraction reagents is more than milliliter, the soluble amount of extraction reagents used in the microfluidic chip can be reduced to microliter, which can extract target molecules from fewer samples, and improve the extraction efficiency by enhancing the mixing between the two phases. It reduces the demand for solvents and reduces the secondary pollution of heavy metals to the environment, which is of great significance to enhance the analysis and detection effect and promote the development of micro detection devices and instruments [5]. Guo et al. believe that microfluidic is a scientific technology based on the theory of non-Newtonian fluid, low Reynolds number laminar flow, multi physical field coupling effect and interface effect, which is mainly characterized by the manipulation of fluid in micron scale space and takes the fluid transport in micro scale as the platform [6]. At present, it has been widely used in medicine, bioengineering, aerospace, and other fields. Multiphase laminar flow extraction in microfluidic chip is a typical technology with microsystem characteristics. Tanataweethum et al. believe that the so-called “micro scale” is not strictly defined, but a concept of relative size. At present, there is no unified formulation on the division of scale. Generally, the scale greater than 1 mm is called macro scale, and the scale of 1 um-1 mm is called micro scale [7]. Kimet al. found that the configuration of the microfluidic liquid-liquid extraction chip channel usually adopts double *Y*-type two-phase laminar flow or double type three-phase laminar flow. The substrate of microfluidic chip is a glass or quartz material resistant to organic solvent, and the microfluidic chip is PDMS organic polymer material [8]. Ulkir et al. tried laminar liquid-liquid extraction based on ion extraction on the microfluidic chip. They independently introduced the organic solution containing neutral ion carrier and lipophilic pH indicator dye and the aqueous solution containing sample ions into the microchannel to form an oil-water interface. After the organic phase and aqueous phase formed a stable laminar flow, the selective extraction of a variety of ions was realized based on the selective difference between the ions of neutral ion carrier and the extract. Then, the ions were measured downstream of the organic phase by thermal lens microscope under continuous flow conditions [9]. Subsequently, Ahmed et al. constructed a three-phase flow microfluidic extraction device in the microchannel (150 *μ*m × 25 *μ*m) on the glass microchip (3 cm × 7 cm) and used it as a liquid membrane to separate the spontaneous phase separation of the three-phase flow in the microfluidic device caused by the surface modification of the microchannel by octadecylsilane groups. The three-phase flow in the microchannel was used as a liquid membrane to observe the selective transport of ions through the liquid membrane. As a result, a selective separation device from the target metal ion from the aqueous feed solution to the receiving phase in a few seconds [10]. Zhao et al. designed and manufactured microfluidic chips based on reverse laminar flow. In order to produce reverse flow of aqueous phase and organic phase, we selectively modified the lower part of microchannel wall with hydrophobic groups, while the upper part remained hydrophilic. In the experiment, the organic phase was introduced into the lower part and the aqueous phase was introduced into the upper part. The velocity ratio between the two phases was studied, and the wide operation range of countercurrent was verified. The results show that the efficiency of one-time reverse parallel extraction using this method is 4-5 times that of left and right parallel extraction [11].

Based on this research foundation, this paper combines the main pollution of heavy metals and the main means of controlling heavy metals in China with microfluidic technology, uses microfluidic technology to extract heavy metal copper, and studies the multiphase laminar flow membrane-free liquid-liquid extraction and membrane-free separation technology of microfluidic chip.

## 3. Research Methods

### 3.1. Microfluidic Liquid-Liquid Extraction Technology

Microfluidic chip (also known as lab-on-a-chip) is the main platform for microfluidic technology operation. The common ways to generate droplets in microfluidic chips include extrusion flow, confocal flow, and coaxial tube flow. Due to the scale effect in the microchannel, the generated droplets have a strong size effect. According to the generation mode of droplets, they can be divided into extrusion flow, confocal flow, and coaxial pipe flow. The oil phase is used as the organic phase and the water phase is used as the water phase [12].

Among them, the t-channel generation of droplets is a traditional droplet generation method. At the two-phase contact interface, droplets are generated through the shear force of the organic phase and the pressure difference before and after the droplets [13]. This method is easy to make and control and is widely used in occasions with low requirements for droplet size, but the controllable flow rate range of droplets generated by this method is small.

### 3.2. Multiphase Laminar Mass Transfer Mechanism in Microchannel

In the traditional liquid-liquid extraction, the organic phase and aqueous phase are layered up and down by using the difference of their density, but others pointed out through theoretical derivation and experimental observation that in the micron channel, the gravity effect caused by the difference of relative surface tension and density between the two phases can be ignored [14]. The theoretical derivation is as follows:

Depth and width of the separation channel, respectively, then the depth width ratio of the microchannel can be expressed as formula (1) by *R*_*dw*_ as follows:

(1) $$\begin{array}{c} R_{dw}=\frac{d}{w}\;. \end{array}$$

Assuming that the organic phase and the aqueous phase each account for half of the channel width, the surface tension and the gravity difference between the two phases can be expressed as 2*γ*(*L*+*d*) and *VρdwLg*/2, respectively [15]. Here, *γ* and Δ*p* are the dimensionless exponent *R*_*g*−*t*_ representing the ratio of gravity to surface tension, and its expression is:

(2) $$\begin{array}{c} R_{g-t}=\frac{V\rho dwLg/2}{2\gamma \left(L+d\right)}. \end{array}$$

Since *L*〉〉*d*, the above formula can be simplified to:

(3) $$\begin{array}{c} R_{g-t}=\frac{V\rho dwg}{4\gamma }. \end{array}$$

Substitute *R*_*dw*_ into the above formula, then *R*_*g*−*t*_ can be expressed as:

(4) $$\begin{array}{c} R_{g-t}=R_{dw}\frac{V\rho g}{4\gamma }w^{2}. \end{array}$$

Under the fixed aspect ratio, that is, *R*_*dw*_ is certain, but for a specific extractant, *γ* and Δ*p* between water are certain values, so *R*_*g*−*t*_ is directly proportional to *w*^2^. Combining the fixed factors *R*_*dw*_*γ* and Δ*p* , expressed by the constant *c*, can be simplified to:

(5) $$\begin{array}{c} R_{g-t}=cw^{2}. \end{array}$$

It can be seen that in microchannels less than 1 mm, the contribution of gravity is much less than the surface tension [16]. At lower flow rates, the aqueous phase and organic phase form a stable laminar flow state without stratification up and down due to different specific gravity. Generally, the formation of laminar flow is that the viscous force of the fluid is much greater than the inertial force of the fluid [17]. In microchannels, laminar flow is usually represented by Reynolds number (*R*_*e*_) as follows.

(6) $$\begin{array}{c} R_{e}=\frac{\rho vD}{\mu }, \end{array}$$

where: *ρ* represents the density of the liquid; *v* is the flow rate of the fluid; *D* represents the size of the pipe diameter; *μ* is the viscosity of the fluid.

It is generally believed that the fluid flow in the microchannel is laminar at a small Reynolds number. Most of the mixing of fluids comes from lateral diffusion. This phenomenon also exists on the traditional scale, but it is not obvious on the macro scale. The diffusion distance (*l*) in one dimension can be expressed as follows:

(7) $$\begin{array}{c} l^{2}=t*D, \end{array}$$

where: *D* represents diffusion coefficient and *t* represents diffusion time. The diffusion distance (*l*) under two-dimensional conditions can be expressed as follows:

(8) $$\begin{array}{c} l^{2}=2t*D. \end{array}$$

The diffusion coefficient *D* is related to the properties of the diffuser itself, which is defined as follow:

(9) $$\begin{array}{c} D=\frac{k_{\beta }T}{6\pi \eta a}, \end{array}$$

where: *T* is the temperature, *η* is the solution viscosity, *k*_*β*_ is the Boltzmann's constant, and *a* is the radius.

### 3.3. Mass Transfer and Diffusion Model of Membrane Free Liquid-Liquid Microextraction

This paper takes double *Y*-type microfluidic as the basic research, adds a microfluidic chip whose inlet becomes double *ψ* -type, takes double *Y*-type and double *ψ* -type microfluidic chips as the model, and its structural dimensions are shown in Table 1.

For the liquid flow in micro scale channel, the continuous flow microfluidic technology of homogeneous system was first developed [18]. Because the flow characteristic scale is in the micron level or even smaller, at this time, it is necessary to reduce the macro horizontal flow size in equal proportion and make use of the characteristics of strengthening mass and heat transfer and reducing reagent consumption brought by the confined space of the micro flow channel to enhance the conversion efficiency and improve the selection function. At this time, the inertial force and gravity of the fluid can be gradually ignored and replaced by the enhancement of viscous shear force and surface tension.

### 3.4. Effect of Auxiliary Structure in Channel on Liquid-Liquid Extraction

In addition, the inlet flow rate will also affect the liquid-liquid extraction of the microfluidic chip. In this paper, the influence of the auxiliary structure added in the channel on the flow field of the micro channel in the actual working process is fully considered. By designing and comparing the influence law of the auxiliary structure on the flow field characteristics in the micro channel, the mixing between the liquid-phase flow layers is enhanced and the efficiency of laminar liquid-liquid micro grass is improved [19]. By analyzing the effects of two-phase inlet velocity, two-phase contact time, two-phase contact interface, and microchannel length on liquid-liquid extraction of microfluidic chip, the reasonable selection range of inlet velocity, contact time, contact interface, and microchannel length in micro scale is summarized. At the same time, the flow characteristics of different polar fluids in microchannel, the mass transfer characteristics of multiphase laminar flow in double *Y*-shaped microchannel, and the influence of channel structure on microscale flow and mass transfer characteristics are analyzed. Based on microfluidic dynamics, the grass extraction efficiency of liquid-liquid microextraction is further explored [20].

In this paper, the double *y* microfluidic chip is taken as the basic research. The cross auxiliary structure, cylindrical auxiliary structure (symmetrical/asymmetric), and the number of shelf inlets are added to this type of microfluidic chip to change the inlet structure into a double *ψ* microfluidic chip and increase the two-phase contact interface.

In microfluidic chip extraction, the corresponding experimental rules are obtained by comparing the effects of different experimental conditions on the extraction efficiency of copper ions [21].

Extraction efficiency *E*_1_ is the percentage of the amount of metal ions in the aqueous phase taken into the organic phase and the total amount of metal ions in the aqueous phase, as shown in the following formula:

(10) $$\begin{array}{c} E=\frac{C_{aq,\text{in}}-C_{ag,\text{out}}}{C_{aq,\text{in}}}\times 100\%. \end{array}$$

In formula (10), *C*_*aq*,in_ represents the concentration of metal ions in the aqueous phase before two-phase contact, and *C*_*ag*,out_ represents the concentration of metal ions in the aqueous phase at the outlet after two-phase contact [22].

In this paper, the extraction efficiency is predicted by the diffusion efficiency *D*. The diffusion efficiency represents the diffusion of copper ions in the aqueous phase to the organic phase, as shown in the following formula:

(11) $$\begin{array}{c} E_{2}=\frac{v_{\text{org }}\cdot t\cdot C_{\text{org,out}}}{v_{aq\;}\cdot t\cdot C_{aq,\text{in}}}\times 100\%=\frac{v_{\text{org}}\cdot C_{\text{org},\text{out}}}{v_{aq\;}\cdot C_{aq,\text{in}}}\times 100\%\;. \end{array}$$

In formula (11), *C*_*aq*,in_ represents the initial analyte concentration at the inlet of the aqueous phase before the simulated two-phase contact, and *C*_org,out_ represents the analyte concentration at the outlet of the organic phase after the simulated two-phase contact.

When the aqueous phase and organic phase are injected into the microfluidic chip at the same flow rate, formula (11) can be rewritten as follows:

(12) $$\begin{array}{c} E_{2}=\frac{C_{\text{org},\text{out}}}{C_{aq,\text{in}}}\times 100\%. \end{array}$$

Finally, by comparing the similarity between *E*_1_ and *E*_2_, it is verified that the higher the diffusion efficiency of two-phase flow, the better the liquid-liquid extraction efficiency of two-phase laminar flow in the experiment [23].

## 4. Result Analysis

### 4.1. Effect of Flow Rate on Diffusion Efficiency

Corresponding mixing comparison experiment: the upper part is the organic phase and the lower part is the aqueous phase added with blue reagent to verify the mixing of oil-water in the two phases. When the inlet velocity is 10^−3^*m*/*s* , the two phases have an obvious phase interface at the intersection of *Y*-shaped inlet, the molecular diffusion distance in the vertical flow direction is short, and the diffusion degree of target molecules from aqueous phase to organic phase increases gradually along the flow direction. When the inlet velocity decreases to 10^−5^ m/s, the diffusion degree of target molecules from aqueous phase to organic plant increases gradually along the flow direction [24].

The molecular diffusion efficiency at different stages is shown in Figure 2: the material diffusion along the flow direction is gradually increasing, and the concentration diffusion at low flow rate is significantly higher than that at high flow rate. When the channel length *L* ≤ 10 mm, the diffusion efficiency of inlet velocity 10^−3^ m/s is about 20%; The diffusion efficiency of inlet velocity 10^−4^ m/s is about 60%, and the concentration diffusion efficiency can reach 95% when the inlet velocity is 10^−5^ m/s and 10^−6^ m/s. This is because under ideal conditions, the lower the speed, the longer the two-phase contact time, the higher the intensity of diffusion efficiency between two-phase molecules, the more sufficient mixing and the higher the extraction efficiency. When the channel length *L* ≤ 30 mm, the diffusion efficiency of inlet velocity 10^−3^ m/s gradually increases to about 45%; the diffusion efficiency of inlet velocity 10^−4^ m/s gradually increases to about 80%; the concentration diffusion tends to be stable at inlet velocity 10^−5^ m/s and 10^−6^ m/s, both of which are about 95%. Therefore, when the velocity is further reduced, the diffusion efficiency can still be maintained at about 95%. Therefore, if the inlet speed is 10^−5^ m/s, it can be selected as the minimum inlet speed of smooth channel [25].

### 4.2. Effect of the Same Flow Rate on Extraction Efficiency

Taking double *Y*-type and double *ψ*-type microfluidic chips as examples, the microchannel length is 30 mm, and the given inlet flow rates are 10^−4^ m/s and 10^−3^ m/s, respectively. The comparison of grass extraction efficiency through the experiment is shown in Figure 3; the extraction efficiency of double *ψ* type was higher than that of double *Y*-type; at the bottom flow rate, the extraction efficiency is low, and when the flow rate increases to 10^−3^ m/s , the extraction efficiency is improved. Based on experiments and numerical simulation, at the bottom flow rate, the aqueous phases of double *Y*-type and double *ψ*-type are broken. Although the two-phase contact interface increases under the same volume, compared with laminar flow, the two-phase contact interface decreases. When the flow rate increases to 10^−3^ m/s , the double *Y*-type and double *ψ*-type aqueous phases show laminar flow, and the two-phase contact interface increases compared with the bottom flow rate, so the extraction efficiency is improved.

### 4.3. Effects of Different Flow Rates on Extraction Efficiency

Taking double *Y*-type and double *ψ*-type microfluidic chips as examples, when the microchannel length is 30 mm and the flow rate of fixed organic phase is *v*_oil_=10^−3^ m/s , the flow rate of changing aqueous phase is half and five times that of organic phase. The comparison of extraction efficiency through experiment is shown in Figure 4; the extraction efficiency of double *ψ*-type is higher than that of double *Y*-type; when the flow velocity ratio increases from *v*_*aq*_ : *v*_oil_=1 : 2 to *v*_*aq*_ : *v*_oil_=5 : 1, the extraction efficiency increases slightly, which may be due to the stable laminar flow state of both aqueous phase and organic phase under this flow velocity ratio, and the change of the width of aqueous phase in the microchannel has no obvious effect on the extraction efficiency. It is confirmed that the two-phase contact interface is the main factor affecting the extraction efficiency.

### 4.4. Effects of Different Auxiliary Structures on Extraction Efficiency

The extraction efficiency of conventional oscillation method and chips with different microchannel structures are comprehensively compared. The results are shown in Figure 5: when the contact time is 15 s, the extraction efficiency of optical channel microfluidic chip is about 1.3–1.6 times that of conventional oscillation; the extraction efficiency of microchannel with a cross auxiliary structure is 1.2–1.5 times that of conventional extraction because the effective contact interface is smaller than that of the optical channel; the extraction efficiency of microfluidic chip with a cylindrical auxiliary structure is 1.5–1.9 times that of conventional extraction. It can be seen that the extraction efficiency of microfluidic chip is higher than that of conventional extraction. For microfluidic chips, the extraction efficiency of cylindrical auxiliary structure is 1.1–1.5 times higher than that of the optical channel. However, there is a large gap between the maximum and minimum extraction efficiency of the cross micro auxiliary structure, and there is no stability of optical channel. The possible reason is that the cross auxiliary structure plays a role in separating two phases rather than mixing two phases in the middle of micro channel. It can be seen that when the two-phase contact time is given, the reasonable design of cylindrical auxiliary structure can make the flow in microchannel more disordered, promote two-phase mixing, effectively improve the molecular diffusion efficiency between multiphase flows, and effectively improve the extraction efficiency of microfluidic liquid-liquid extraction.

Taking the cross and cylindrical micro auxiliary structures as examples, when the microchannel length is 30 mm, the given inlet flow rate is 10^−3^ m/s and the contact time is 15 s, the experimental extraction efficiency is compared with the diffusion efficiency simulated by simulation: the diffusion efficiency of cross and cylindrical is higher than that of extraction efficiency, in which the diffusion efficiency of cross is 1.05 times that of extraction efficiency and that of cylindrical is 1.04 times that of extraction efficiency. The error analysis shows that the reason why the diffusion efficiency is higher than the extraction efficiency is that the diffusion efficiency is the numerical calculation result under ideal conditions, while the extraction efficiency is slightly lower than the diffusion efficiency due to the influence of experimental environment, temperature, and humidity. It can be seen that the numerical calculation method is used to predict the actual diffusion efficiency in the process of liquid-liquid microextraction, and the results have good reliability and stability.

## 5. Conclusion

Based on the theory of microfluidic dynamics, the microfluidic chip is fabricated to reduce the influence of roughness as much as possible. Under the condition that the accuracy can reach 2 um, the equilibrium time of reaction is shortened and the extraction efficiency is improved. Compared with the conventional extraction experiments, the effect of microfluidic technology on the extraction and separation of copper was also studied. Among them, the effects of inlet flow rate and contact time on liquid-liquid extraction of copper were studied in double *Y* microfluidic chip. Compared with double *ψ* microfluidic chip, the effects of contact interface on liquid-liquid extraction of copper were studied, and the following conclusions were drawn:

1. Taking the double *Y*-type liquid-liquid extraction microfluidic chip as the research object, this paper analyzes the diffusion and mass transfer process of copper ion from water phase to extractant oil phase in microchannel. Through the combination of numerical analysis and experiment, the relationship between copper ion flow law and extraction efficiency in the microchannel is analyzed. It is found that the mass transfer interface caused by the concentration difference between aqueous phase and organic phase in the microchannel is not located in the center of the channel, but related to the physical properties such as the viscosity of the working medium liquid.
2. Through the design and addition of auxiliary structure, it is confirmed that the auxiliary structure can increase and strengthen the mass transfer at the two-phase contact interface and improve the liquid-liquid extraction efficiency. In this paper, double *ψ*-type microfluidic chip is introduced to confirm the relationship between the contact interface and the extraction efficiency. On the one hand, the increase of contact interface improves the extraction efficiency, but not in a positive proportion; on the other hand, the addition of auxiliary structure can increase the disturbance degree of fluid in the microchannel, change the local stress and promote the two-phase mass transfer. In this paper, the extraction efficiency of metal ions and the service life of the chip can be rapidly improved by selecting the appropriate microchannel structure and inlet flow rate. It has important theoretical and practical guiding value for the extraction of rare and valuable materials containing complex impurities or low content.

## Figures and Tables

**Figure 1:** Droplet microfluidic two droplet preparation system.

**Figure 2:** Diffusion efficiency at different inlet velocities.

**Figure 3:** Comparison of extraction efficiency of different types of microfluidic chips under the same flow rate ratio.

**Figure 4:** Comparison of extraction efficiency of different types of microfluidic chips under different flow rate ratio.

**Figure 5:** Extraction efficiency under different extraction methods.

**Table 1:** Structural dimension parameters of different internal structures of microfluidic chip (unit: um).

Characteristic symbol	Double *Y*-shaped optical channel	Dual *ψ*-type optical channel
*L*_1_	30000	30000
*h*_1_	120	120
*W*_1_	600	600

## Data Availability

The data used to support the findings of this study are available from the corresponding author upon request.
